# Study on Management of Blood Transfusion Therapy in Patients with Hereditary Spherocytosis

**DOI:** 10.1155/2022/6228965

**Published:** 2022-01-28

**Authors:** Shiyue Ma, Lingjian Tang, Chaoli Wu, Hui Tang, Xue Pu, Jinhong Niu

**Affiliations:** ^1^Department of Laboratory Medicine, Affiliated Hospital of Guilin Medical University, Guilin City 541001, Guangxi Zhuang Autonomous Region, China; ^2^Department of Rehabilitation Medicine, Affiliated Hospital of Guilin Medical University, Guilin City 541001, Guangxi Zhuang Autonomous Region, China; ^3^Department of Medical Administration, Nanxishan Hospital of Guangxi Zhuang Autonomous Region, Guilin City 541002, Guangxi Zhuang Autonomous Region, China

## Abstract

Hereditary spherocytosis (HS) is a chronic hemolytic disorder caused by inherited defects in the red blood cell membrane. This study discusses the treatment strategy for the decline in hemoglobin level in three HS probands with moderately severe or severe hemolysis and summarizes the appropriate laboratory tests that help improve clinical management of blood transfusion in HS patients. Three probands who were diagnosed with HS in our hospital and their family members were included in this study. Clinical data of the three families were reviewed to summarize their hematopoietic characteristics. DNA from all family members of the 3 HS probands was amplified by polymerase chain reaction (PCR) and sequenced by the Sanger method to assess genetic relation for HS. Based on the sequencing results, the type of mutated membrane protein in each proband was analyzed using the eosin-5′-maleimide (EMA) binding test and sodium dodecyl sulfate polyacrylamide gel electrophoresis (SDS-PAGE). The hemoglobin level was reduced in all 3 probands after different levels of infection. The fluorescence of EMA-labeled red blood cell (RBC) was decreased. DNA sequencing showed that His54Pro, Leu1858Val, and 6531-12C>T compound heterozygous mutations were present in the *SPTA1* gene of patient I-1, Arg344Gln and c.609+86G>A heterozygous mutations were present in the *SLC4A1* gene of patient II-1, and Leu2032Pro homozygous mutation was present in the *SPTB* gene of patient III-1. SDS-PAGE results demonstrated that the concentration of band 3 was reduced in II-1, whereas the levels of the corresponding mutant proteins in the other probands were unchanged. The family members of the respective patients presented mutations in major genes causing HS. The Leu2032Pro mutation identified in patient III-1 is a new missense mutation of the *SPTB* gene in the Chinese population that has never been reported in literature previously. The presence or absence of acute or chronic infections is a critical deciding factor for the treatment and clinical management of HS patient via blood transfusion. For patients with infections, hemoglobin concentration can be restored once the infection is controlled, thus obviating the need for proper infection control before blood transfusion.

## 1. Introduction

Hereditary spherocytosis (HS) is a hereditary hemolytic anemia caused by abnormalities in the red blood cell (RBC) membrane proteins. About 75% patients have autosomal dominant HS and 25% have autosomal recessive or newly mutated HS [1, 2]. It is currently the most prevalent type of hemolytic anemia among inherited RBC membrane disorders and is widespread across the different races. The incidence rate of HS can be as high as 1/10000-1/2000 in northern Europe [3]. Despite the lack of accurate epidemiological statistics, HS is not an uncommon disease in China as it can be found in about 1.27 males and 1.49 females per 100,000 [4, 5]. The typical clinical manifestations of HS are anemia, jaundice, splenomegaly, high spherocyte load in blood smear, increased RBC osmotic fragility, and chronic anemia accompanied by acute hemolysis [6]. HS can be classified as mild, moderate, moderately severe, and severe based on various clinical parameters such as hemoglobin (Hb) levels, reticulocyte count, bilirubin, peripheral smear, splenectomy [7], and transfusion [2]. Hemolytic crisis is most common in severe HS patients and presents with fever that may be triggered by viral infections [8]. Most patients are autosomal dominant for HS with a clear family history of the disease. The type of HS-causing gene mutations differs across different races and populations [9]. Patients with severe HS often need to rely on blood transfusions in order to maintain their Hb levels at 60 g/l. On the other hand, patients with moderately severe HS may require intermittent blood transfusions to prevent dramatic reduction in Hb level leading to fatigue and infection [10]. However, long-term chronic transfusion may easily lead to iron overload, resulting in deposition of iron in various organs and tissue parenchymal cells and consequently organ failure [11].

Given that HS patients have diverse clinical manifestations and are treated sporadically, the disease is often overlooked by the clinicians, resulting in misdiagnosis or missed diagnosis. Furthermore, studies on the treatment of HS patients with infections and critically low Hb levels are still lacking. In this study, we report the diagnosis and clinical laboratory pattern of three HS patients. The HS patients were diagnosed on the basis of blood tests and other laboratory findings. We also evaluated the effect of concurrent infection treatment on its consequences on Hb level and blood transfusion. Moreover, we also examined the types of mutated genes and proteins in three unrelated moderately severe or severe HS probands and their families and summarized the relevant blood transfusion measures that were taken during their treatment.

## 2. Materials and Methods

This study was approved by the Ethics Committee of the First Affiliated Hospital of Guangxi Medical University, and written informed consent was obtained from all subjects and their legal guardians. All the reagents and chemicals used in this research were of high purity. Eosin-5′-maleimide (EMA) powder was purchased from the Sigma-Aldrich Company, Poole, Dorset, UK. Full automatic biochemical instrument (Model 7600, Hitachi, Tokyo, Japan) was used for liver function tests. An automated hematology analyzer (Model LH 780; Beckman Coulter, California, USA) was used for routine blood examination. Fetal bovine serum (FBS) was acquired from Life Technologies Corporation, Shanghai, China. DNA extraction was performed using an omega kit (Omega Bio-Tek Inc., Copenhagen, Denmark). PCR amplification was conducted in the T100 Thermal Cycler (Bio-Rad, California, USA). DNA Purification Kits were purchased from Solarbio Life Science, Shanghai, China. A broad range unstained protein marker was obtained from Tiangen Biotech Co., Ltd., Beijing, China. Detailed procedure for each process is given below.

### 2.1. Specimen Collection and Routine Laboratory Examination

All probands were diagnosed with HS according to the ICSH guidelines [12]. Intravenous blood samples were collected (with one tube for EDTA-K2 anticoagulation and one tube for separation gel coagulation). Liver function, especially total bilirubin (TBIL) and direct bilirubin (DBIL), was performed using a 7600 full automatic biochemical instrument (Hitachi, Tokyo, Japan), and an LH 780 automated hematology analyzer (Beckman Coulter, California, USA) was used for blood routine examination. Spherocytosis in the peripheral blood was stained with Wright's staining, and the cells' morphological examination and number counting were rechecked with an ordinary microscope. Five hundred red blood cells were evaluated in each blood smear for the percentage of spherical red cells, and red cells with other shape abnormalities. The guidelines for the standardization of peripheral blood smear interpretation were from the Chinese Journal of Laboratory Diagnosis.

### 2.2. Eosin-5′-Maleimide (EMA) Binding Test

The eosin-5′-maleimide (EMA) binding test is currently the most sensitive, specific, and convenient diagnostic test for HS. The modification of the method described by Park et al. [13] was used for this test. Briefly, 500 *μ*l of EDTA-K2 anticoagulated blood was collected from the HS probands and non-HS probands and washed 3 times in 1.5 ml phosphate-buffered saline (PBS) at 2500 rpm for 5 min each. Eosin-5′-maleimide (EMA) powder (Sigma-Aldrich Company, Poole, Dorset, UK) was dissolved in PBS to a final concentration of 0.5 mg/ml, stored at -20°C, and thawed at 4°C prior to use. The washed RBCs (5 *μ*l) were resuspended in 25 *μ*l EMA dye, and the mixture was incubated at room temperature for 1 h in the dark, followed by washing 3 times in PBS containing 0.5% fetal bovine serum (Life Technologies Corporation, Shanghai, China) at 2500 rpm for 5 min each. After decanting the supernatant, the pellet was resuspended in 600 *μ*l PBS. The cells were acquired on BD Accuri® C6 (Becton Dickinson company, San Jose, CA), and the MFI (mean fluorescence intensity) value was determined for 15,000 events in the FL1 channel and analyzed with BD FACSDiva software. RBCs emit green fluorescence when they bind EMA. In order to reduce the intra-assay error in measurement, probands' and their families' samples were compared with simultaneously acquired six controls per test run [14]. Parameters of EMA binding tests were expressed as EMA (%), the percentage of the EMA binding values (MFIs) of the proband's RBCs relative to those of the normal controls.

### 2.3. Polymerase Chain Reaction and DNA Sequencing

Peripheral blood genomic DNA was extracted from the probands and their family members using the omega kit (Omega Bio-Tek Inc., Copenhagen, Denmark). Primers for the *SPTA1*, *SPTB*, *ANK1*, *SLC4A1*, and *EPB42* genes, including their exons and adjacent introns, were designed using the Primer Premier 5.0 software (Beijing Genomics Institute; China). PCR amplification was conducted in the T100 Thermal Cycler (Bio-Rad, California, USA) using the following reaction mixture and cycling conditions: 25 *μ*l PCR Master Mix (Takara Bio, Otsu, Japan), 1 *μ*l forward primer, 1 *μ*l reverse primer, 0.2 ng DNA, and double distilled water in a 50 *μ*l total reaction volume; 95°C predenaturation for 5 min, followed by 35 cycles of denaturation at 95°C for 30s, annealing at the suitable temperature for primer set for 30 s and extension at 72°C for 4 s, and concluded by a final extension at 72°C for 8 min and 4°C hold. The PCR products were run in a 1.5% agarose gel, and the target amplicons were purified using the DNA Purification Kit (Solarbio Life Science, Shanghai, China) and sequenced by the ABI 3730xl sequencer (Applied Biosystems, New York, USA).

### 2.4. Preparation and Analysis of Erythrocyte Membranes

Erythrocyte membranes were prepared from the peripheral blood according to the previously described procedure [15] except that 1 mM phenylmethylsulfonyl fluoride was added during the lysis step. Loading buffer (containing *β*-mercaptoethanol) was added to the erythrocyte membrane protein. Then, the mixture was kept in 37°C for 40 min and analyzed by sodium dodecyl sulfate polyacrylamide gel electrophoresis (SDS-PAGE) in a 3.5%-17% linear gradient of acrylamide monomer according to Fairbanks et al. [16]. Broad range unstained protein marker (Tiangen Biotech Co., Ltd., Beijing, China) was used to indicate the molecular weight of protein. Gels were stained with Coomassie blue and scanned by the Gel Doc 2000 Imaging system (Bio-Rad company, California, USA). Protein content was expressed as a ratio to corresponding health controls.

## 3. Results

### 3.1. Patient and Routine Blood Tests

The blood and liver function test results of all the three probands and their families were carried out, and their results are shown in Table 1. Neither of the 3 probands had any consanguineous marriage.

In family 1, the proband was a 9-year-old boy (I-1) diagnosed with neonatal hyperbilirubinemia without exchange transfusion at birth. At 4 months of age, the I-1 appeared pale and dispirited without apparent cause and was not diagnosed with HS at that time. At 2 years of age, I-1 was admitted to the local hospital due to bronchopneumonia and 3 days of fever. Relevant laboratory tests showed 2.64 × 10^12^ RBCs/l and 54 g/l Hb. Although administration of cough suppressant and antipyretic medications did not improve his condition, antiviral and anti-infective therapy restored his body temperature to normal and ceased his coughing. Routine blood test revealed mild anemia, but blood transfusion was not required. However, the anemia exacerbated over time, and he became transfusion-dependent requiring an average 1-2 transfusions per month. At that stage, the cause of disease had still not been identified. When the proband turned 9, he was admitted to our hospital with a history of “2 days of fever” and indicated no history of hereditary disease. Routine blood tests showed 45.9 g/l Hb, 3503 ng/ml serum iron, and 25% spherocytes (Figure 1). Based on his medical history, clinical symptoms, and laboratory test results, the proband was diagnosed with severe HS. No significant abnormalities were observed in the proband's father (I-2) and mother (I-3). After completion of relevant tests and preoperative preparations, the proband underwent splenectomy, and in the duration between admission and splenectomy, his Hb levels dropped to 30 g/l due to acute upper respiratory tract infection. An anti-infective and cough treatment restored the levels to 51 g/l, and therefore, blood transfusion was not given to the proband.

In family 2, the proband was a 7-year-old girl (II-1) whose clinical characteristics were normal until she had acute tonsillitis. She was admitted in our hospital with fever and jaundice, and routine testing showed her Hb level of 53.6 g/l. Tests for urine, kidney function, electrolyte, cardiac enzyme, and coagulation were all normal. II-1 was finally diagnosed with HS after screening through a series of hemolytic indices which showed 15% spherocytes in her blood. After cefmetazole anti-infective therapy, she no longer had fever and sore throat, and her jaundice had also subsided. Her Hb level was increased to 74.4 g/l, and she was not given any blood transfusion during treatment. There was no family history of jaundice or anemia tendency.

In family 3, the proband was an 18-month-old boy (III-1) who was admitted to the hospital due to fever and acute pharyngitis. He was pale at birth but had no other clinical symptoms. He was not diagnosed with HS at that time and was not given any treatment apart from iron supplements. The proband was diagnosed with HS only after comprehensive testing at our hospital. His test results indicated 48 g/l Hb and 28% spherocytes, and his Hb level was increased to 62 g/l after anti-infective and detoxification therapy. The proband's mother (III-3) had mild anemia, whereas the father (III-2) had normal laboratory test results.

### 3.2. The Eosin-5′-Maleimide (EMA) Binding Test of Probands and Normal Controls

The flow cytometric analysis of EMA-labelled erythrocytes revealed, in the probands (Figure 2), that the fluorescence peaks were shifted to the left, and a 35.77%, 24.97%, and 20.64% reduction of the intact erythrocyte fluorescence intensity corresponding to (I-1), (II-1), and (III-1) when compared with normal controls in the each term.

### 3.3. Genetic Analysis

We screened for the *SPTA1*, *SPTB*, *ANK1*, *SLC4A1*, and *EPB42* mutations in the probands and their families using PCR followed by Sanger sequence analysis. In family 1, the DNA sequencing of the proband (I-1) revealed compound heterozygous mutations in *SPTA1* (Figure 3). The mutations consisted of the following: a heterozygous mutation c.161A>C in exon 2, which resulted in a His^54^>Pro^54^ substitution in *α*-spectrin, a novel mutation. A heterozygous mutation c.5572C>G in exon 40, which resulted in Leu^1858^>Val^1858^ and a heterozygous mutation 6531-12C>T in intron 45. Based on DNA sequence analysis, Leu1858Val and 6531-12C>T were found to be inherited from the proband's father (I-2), and His54Pro was found to be inherited from the proband's mother (I-3).

In family 2, the two heterozygous mutations were found in *SLC4A1* from the proband (II-1), one was missense mutation c.1031G>A in exon 9, which resulted in a Arg^344^>Gln^344^ substitution in band 3. The other was a heterozygous mutation c.609+86G>A in intron 7. Family members were verified according to these mutation sites; data suggested that Arg344Gln was identified in the mother (II-3) and brother (II-4); c.609+86G>A was identified in the father (II-2).

In family 3, a homozygous c.6005T>C in exon 29 of *SPTB* was identified in the proband (III-1), resulting in a Leu^2032^>Pro^2032^ substitution in *β*-spectrin, a novel mutation. A heterozygous form of Leu2032Pro was found in both the father (III-2) and the mother (III-3).

### 3.4. Sodium Dodecyl Sulfate Polyacrylamide Gel Electrophoresis

Following the DNA sequence results of the mutant gene, we investigated the level of this genetic alteration on the probands' red-cell membrane. Densitometry of Coomassie blue stained SDS-PAGE of erythrocyte membrane proteins was used to quantify the content of relative protein that expressed the mutated gene and the mutated protein/healthy protein relation used to calculate the abnormal-associated protein content (Figure 4). By this method, proband I and proband III presented an indiscrimination reduction of *α*-spectrin and *β*-spectrin content, respectively, and proband II presented a 17% reduction of band 3.

## 4. Discussion

Mutations in genes encoding RBC membrane proteins cause HS. Less membrane surface area results from these mutations, leading to spherocytes or RBCs. For this reason, phagocytes readily take them up in the splenic microcirculation, resulting in extravascular hemolysis. The predominant pathogenic RBC proteins associated with HS include *α*-spectrin (*SPTA1*), *β*-spectrin (*SPTB*), ankyrin (*ANK1*), band 3 (*SLC4A1*), and protein 4.2 (*EPB42*). In addition, approximately 1% of HS patients carry Rh complex defects as well [17].

RBC morphology and RBC osmotic fragility tests are currently used to diagnose HS. According to Liao et al., MSCV can distinguish between HS and Thalassemia, which is clinically similar to HS [18]. They also discovered that MSCV combined with RBC morphology and osmotic fragility by flow cytometry can be used to diagnose HS [19, 20]. Xu et al. proposed MRV as a novel parameter for screening HS; an MRV ≤ 95.77 fl has an 86.8% sensitivity and 91.2% specificity for the diagnosis of HS [21]. In our study, all probands had MSCV < MCV and MRV ≤ 95.77 fl, consistent with other reports. Furthermore, routine blood test of II-3 and II-4 indicated MSCV < MCV, suggesting that they are asymptomatic carriers of HS mutations.

Today, the EMA-binding test is the most sensitive, specific, and convenient way to diagnose HS. The International Council for Standardization in Haematology recommends using it in conjunction with other RBC osmotic fragility tests to improve diagnostic sensitivity [12]. EMA binds to the extracellular domain of band 3 protein on the RBC membrane [22]. A subsequent study found that apart from band 3 protein defects, spectrin protein defects can also decrease the fluorescence intensity of the EMA binding test [23]. The three probands in this study showed different levels of reduction in EMA fluorescence, demonstrating that the EMA test is a superior auxiliary examination for the clinical diagnosis of HS [24]. However, it is important to note that EMA fluorescence is not reflective of the severity of HS [25].

Most patients are autosomal dominant for HS with a clear family history of the disease. Although *ANK1*, *SLC4A1*, and *SPTB* gene mutations are most common among HS patients, about 25% of patients have no family history of the disease suggesting new gene mutations, phenotypic variations, or autosomal recessive inheritance usually in the *SPTA1* and *EPB42* genes [26]. The type of HS-causing gene mutations differs across different races and populations [9]. A recent study showed that disease severity in HS patient is associated with the type of mutant membrane protein [27]. Therefore, a clear identification of the mutant membrane protein and a gene mutation profile has significant implications on the diagnosis, treatment, and prognosis of HS [28].

I-1 carried *SPTA1* compound heterozygous mutations, which are found in approximately 5% of HS patients worldwide and are usually inherited as autosomal recessive mutations [2]. The 3 mutations identified in I-1 were His54Pro, Leu1858Val, and 6531-12C>T. Based on the sequencing results of the parents, it was found that the father (I-2) carried the Leu1858Val and 6531-12C>T mutations and the mother (I-3) carried the His54Pro mutation. Leu1858Val and 6531-12C>T constitute the highly frequent but low expression polymorphic allele “*LELY*” [29]. The 6531-12C>T mutation induces codon skipping in 50% of the exon 46 transcript, resulting in the deficiency of 6 amino acids that link *α*-spectrin and *β*-spectrin. On the other hand, the c.5572C>G mutation causes a change in the amino acid and is found to be in linkage disequilibrium with 6531-12C>T. His54Pro is a new mutation that has not yet been included in the NCBI database. Its pathogenesis is unclear and may be related to destabilization of the polypeptide chain caused by a change in amino acid due to base substitution or a change in mRNA expression level. A single *SPTA1* heterozygous mutation or polymorphic “*LELY*” usually does not result in protein defects that lead to severe clinical symptoms in the patients because *α*-spectrin overexpression can maintain intracellular protein levels, and hence, the damage is mild even if these mutations are pathogenic [30]. However, when both mutations were inherited simultaneously by I-1, *α*^LELY^ potentiated the pathogenic role of His54Pro, which in turn exacerbated the trans expression of *α*-spectrin [31], leading to a vicious cycle that resulted in significant hemolysis in I-1.

II-1 had no clear clinical symptoms at birth but was found to have reduced Hb level when she developed tonsillitis. HS was caused by the synergistic effect of a single exon mutation (Arg344Gln) and a single base substitution (c.609+86G>A) in the intron of the *SLC4A1* gene. There is increasing evidence on the pathogenic role of intron mutations of the *SLC4A1* gene in HS. Van Zwieten et al. found that 7 of 15 new mutations in the *SLC4A1* gene in HS patients were intron mutations and these mutations affected the normal synthesis of pre-mRNA of the *SLC4A1* gene [32]. Synergy between the Arg344Gln and c.609+86G>A mutations was the main cause of reduced band 3 protein concentration in proband II-1.

III-1 carried a Leu2032Pro homozygous mutation that caused significant anemia in the proband after birth, accompanied by a substantial decrease in fluorescence in EMA-labeled RBCs. About 20% HS patients have *SPTB* mutations which are inherited in an autosomal dominant manner [33]. In general, heterozygous mutations in the *SPTB* gene have diverse clinical manifestations which predominantly appear as asymptomatic or mild, such as those in III-2 and III-3. Since *β*-spectrin can also be overexpressed, the damage caused by the *trans* form in the patients may be neglected once the *cis* form of *β*-spectrin reaches sufficient levels. In contrast, patients with homozygous mutations often have moderate to severe HS, but they do not require blood transfusion to sustain life, at least not in the first year of birth [34]. The Leu2032Pro mutation identified in this study is a new missense mutation of the *SPTB* gene in the Chinese population that has never been reported in literature previously. We believe that this mutation does not affect the expression level of *β*-spectrin but may change its protein structure, resulting in RBC membrane skeleton dysfunction and consequently significant anemia in III-1.

Because RBC synthesis is reduced in severe HS newborns, appropriate blood transfusions can be performed. The procedure may affect erythropoietin activity and lead to transfusion in HS paediatric patients over 9 months of age and Hb level of 50-60 g/l [1]. Conservative treatment is generally recommended for patients without anemia and jaundice but who have substantially reduced Hb level following infection [35]. We found that II-1, II-3, and II-4 all carried pathogenic gene mutations but given that the clinical symptoms of heterozygous mutations of the band 3 protein are relatively mild as the wild type allele in trans partly compensates for the mutated allele [34], the cause of sudden anemia in II-1 should first be identified before symptomatic treatment is given to the proband.

In patients with severe anemia, missed early HS diagnosis may result in unnecessary blood transfusions [36]. As a result of the misdiagnosis, I-1 was treated late. Before the splenectomy, he received long-term life-sustaining blood transfusions. When the proband experienced acute hemolysis, the new blood transfusion provided I-1 with a significant amount of healthy human RBCs. This may have caused a misdiagnosis due to the proband's high level of RBC debris. Transfusions caused iron overload in I-1, causing liver and heart damage. In addition, multiple blood transfusions can induce the generation of other alloimmune antibodies aside from the ABO blood group system, causing problems in blood cross-matching and clinical treatment and are often greater potential threats than anemia. I-1 had multiple respiratory tract infection-induced anemia and had dramatic reduction in Hb below the indication threshold for blood transfusion. Clinicians from other hospitals often give RBC transfusion before anti-infective therapy. However, we found that anti-infective therapy could alleviate hemolysis in I-1. Any unnecessary transfusion of blood products may not only induce systemic allergy but also increase the risk of infectious diseases [37]. Moreover, transfused RBC may also be subjected to abnormal immune- or non-immune-mediated damage in the patient that will ultimately lead to further hemolysis.

Splenectomy is the most reliable and effective treatment for severe HS [1]. Although this procedure cannot change RBC morphology, it can largely decrease the level of RBC damage and restore the lifespan of RBCs back to near normal, thereby reducing RBC transfusion-dependency in HS patients. If splenectomy is not performed in a timely manner, the patients will experience retarded growth and development and extramedullary hematopoiesis that may progress to Thalassemia [2]. It is important to note that the spleen is an immune organ of the body and early resection of the spleen can increase the risk of infection. The British Committee for Standardization in Haematology recommends splenectomy for individuals >6 years old and recommends subtotal splenectomy over total splenectomy whenever possible. This not only prolongs RBC lifespan but also retains the immune functions of the spleen for at least 5 years [38].

Anemia was quickly ameliorated in I-1 within a year after splenectomy. The proband no longer had jaundice and no longer required long-term blood transfusion for life support. Total iron concentration in the proband was reduced following iron-chelating therapy, resulting in a substantially decreased level of iron toxicity in the liver and heart and significantly enhanced quality of life.

## 5. Conclusion

Hereditary spherocytosis (HS) is a chronic hemolytic disorder caused by inherited defects in the red blood cell membrane. HS has diverse clinical manifestations and is easily misdiagnosed or undiagnosed. If patients with anemia, jaundice, and splenomegaly are identified in clinical settings, further hemolysis-related examinations should be performed. Patients with severe HS often need to rely on blood transfusions in order to maintain their Hb levels at approximately 60 g/l. In addition, patients with moderately severe HS may require intermittent blood transfusions to prevent dramatic reduction in Hb level. However, long-term chronic transfusion may easily lead to iron overload, resulting in deposition of iron in various organs and tissue parenchymal cells and consequently lead to organ failure. For patients that rely on long-term RBC replacement therapy, the pros and cons of blood transfusion should be fully weighed to minimize the number of transfusions and transfusion-induced adverse reactions in order to delay or prevent ineffective RBC transfusion. The presence or absence of acute or chronic infection is very critical to decisions regarding blood transfusion of HS patients. The results of this study showed that infection control in HS patients is a very critical factor to be considered before going for blood transfusion. All the three cases reported in this study restored the Hb level when their infection was controlled and eliminated the need for blood transfusion. Hence, for patients with infections, hemoglobin concentration can be restored once the infection is controlled, thereby precluding blood transfusion.

## Figures and Tables

**Figure 1:** Peripheral blood smear, from top to bottom, I-1, II-1, and III-1, respectively.

**Figure 2:** Flow cytometric evaluation of EMA-labeled red blood cells. Experimental procedure was as described in Materials and Methods. The fluorescence of EMA-stained RBC was obtained for proband I-1 (a), proband II-1 (c), and proband III-1 (e), and their overlay plot compared to the healthy control corresponding to (b), (d), and (f) are shown.

**Figure 3:** DNA sequencing results of proband I-1 (a-1, a-2, a-3), proband II-1 (b-1, b-2), and proband III-1 (c). In the proband I-1, a-1, a-2, and a-3 correspond to His54Pro, Leu1858Val, and 6531-12C>T of *SPTA1*, respectively. In the proband II-1, b-1 and b-2 correspond to Arg344Gln and c.609+86G>A of SLC4A1, respectively. In the proband III-1, homozygous mutation Leu2032Pro is shown in c.

**Figure 4:** SDS-PAGE analysis of erythrocyte membrane proteins using Coomassie brilliant blue staining. Lines I, II, III, and C correspond to erythrocyte membrane proteins from I-1, II-1, III-1, and a healthy control individual, respectively.

**Table 1:** Laboratory characteristics of probands and their families.

Item	RBC (×10^12^/l)	Hb (g/l)	MCV (fl)	MCHC (g/l)	MSCV (fl)	MRV (fl)	Ret (%)	TBIL (*μ*mol/l)	DBIL (*μ*mol/l)
Family 1									
I-1	1.69	45.9	79.69	360.8	75.68	89.30	7.0	178.10	59.20
I-2	4.93	149.2	93.77	322.6	96.38	112.18	1.4	15.60	5.50
I-3	4.80	134.4	85.81	326.1	80.59	106.68	0.9	10.40	3.00

Family 2									
II-1	1.82	53.6	78.33	336.70	67.74	87.65	17.6	48.3	8.7
II-2	6.84	158.40	73.12	316.50	79.14	101.64	7.9	4.40	1.80
II-3	5.04	130.5	81.11	319.50	71.74	95.61	1.4	10.80	3.30
II-4	5.70	168.20	89.17	331.20	87.42	112.53	0.8	8.80	3.50

Family 3									
III-1	1.86	43.0	71.60	326.00	59.14	82.29	12.2	33.50	13.10
III-2	5.17	153.6	91.70	323.80	100.12	117.98	0.8	12.30	4.50
III-3	4.76	120.4	79.70	317.40	88.09	109.70	0.9	17.70	6.00

Abbreviations: RBC: red blood cell count; Hb: hemoglobin; MCV: mean corpuscular volume; MCHC: mean corpuscular hemoglobin concentration; MSCV: mean sphered corpuscular volume; MRV: mean reticulocyte volume; Ret%: reticulocyte ratio%; TBIL: total bilirubin; DBIL: direct bilirubin.

## Data Availability

The data used to support and prove the findings of this study are available from the corresponding author upon request.

## Abbreviations

DBIL: Direct bilirubin
DNA: Deoxyribonucleic acid
EMA: Eosin-5′-maleimide
FBS: Fetal bovine serum
Hb: Hemoglobin
HS: Hereditary spherocytosis
ICHS: International Committee for Standardization of Hematology
MCV: Mean corpuscular volume
MCHC: Mean corpuscular hemoglobin concentration
MSCV: Mean sphered corpuscular volume
MRV: Mean reticulocyte volume
PBS: Phosphate-buffered saline
RBC: Red blood cell
Ret%: Reticulocyte ratio
SDS-PAGE: Sodium dodecyl sulfate polyacrylamide gel electrophoresis
TBIL: Total bilirubin.
